The article "Qualitative Analysis of the Transmission Dynamics of Dengue with the Effect of Memory, Reinfection, and Vaccination" was published in 2022. Journal: Comput Math Methods Med.

# Qualitative Analysis of the Transmission Dynamics of Dengue with the Effect of Memory, Reinfection, and Vaccination

**DOI:** 10.1155/2022/7893570

**Published:** 2022-09-19

**Authors:** Tao-Qian Tang, Rashid Jan, Ebenezer Bonyah, Zahir Shah, Ebraheem Alzahrani

**Affiliations:** ^1^International Intercollegiate Ph.D. Program, National Tsing Hua University, Hsinchu 30013, Taiwan; ^2^Department of Internal Medicine, E-Da Hospital, Kaohsiung 82445, Taiwan; ^3^School of Medicine, College of Medicine, I-Shou University, Kaohsiung 82445, Taiwan; ^4^Department of Family and Community Medicine, E-Da Hospital, Kaohsiung 82445, Taiwan; ^5^Department of Engineering and System Science, National Tsing Hua University, Hsinchu 30013, Taiwan; ^6^Department of Mathematics, University of Swabi, Swabi, 23430 KPK, Pakistan; ^7^Department of Mathematics Education, University of Education Winneba Kumasi (Kumasi Campus), Kumasi 00233, Ghana; ^8^Department of Mathematical Sciences, University of Lakki Marwat, Lakki Marwat, 28420 KPK, Pakistan; ^9^Department of Mathematics, Faculty of Science, King Abdulaziz University, P.O. Box 80203, Jeddah 21589, Saudi Arabia

## Abstract

Dengue fever has a huge impact on people's physical, social, and economic lives in low-income locations worldwide. Researchers use epidemic models to better understand the transmission patterns of dengue fever in order to recommend effective preventative measures and give data for vaccine and treatment development. We use fractional calculus to organise the transmission phenomena of dengue fever, including immunisation, reinfection, therapy, and asymptotic carriers. In addition, we focused our study on the dynamical behavior and qualitative approach of dengue infection. The existence and uniqueness of the solution of the suggested dengue dynamics are inspected through the fixed point theorems of Schaefer and Banach. The Ulam-Hyers stability of the suggested dengue model is established. To illustrate the contribution of the input factors on the system of dengue infection, the solution paths are studied using the Laplace Adomian decomposition approach. Furthermore, numerical simulations are used to show the effects of fractional-order, immunity loss, vaccination, asymptotic fraction, biting rate, and therapy. We have established that asymptomatic carriers, bite rates, and immunity loss rates are all important factors that might make controlling more challenging. The intensity of dengue fever may be controlled by reducing mosquito bite rates, whereas the asymptotic fraction is risky and can transmit the illness to noninfected regions. Vaccination, fractional order, index of memory, and medication can be employed as proper control parameters.

The article "Qualitative Analysis of the Transmission Dynamics of Dengue with the Effect of Memory, Reinfection, and Vaccination" was published in 2022. Journal: Comput Math Methods Med.

## 1. Introduction

Dengue infection is a well-known tropical illness transmitted by female Aedes aegypti mosquitoes and generated by dengue viruses. Due to global warming, dengue disease has extended to approximately 128 nations around the globe, posing a threat to public health and the economy [1]. Dengue virus causes headaches, joint pain, high fever, vomiting, nausea, lower back pain, extreme weakness, muscle pain, rash, bone pain, pain behind the eyes, red eyes, and extreme exhaustion. After sucking blood, the virus is transferred to a mosquito, which then distributes the infection to others. After then, the mosquitoes are diseased for the remainder of their lives, and there have been a few cases of vertical dengue virus transmission [2, 3]. Dengue vaccines have been developed in large part due to the surge in popularity of dengue virus infection in recent decades. Vaccinations against dengue illness are available in some countries [4, 5], but completely effective vaccines have yet to be launched. The researcher proposes several control measures for preventing dengue illness, but additional research is required to develop viable techniques.

It is obvious that mathematical models play an important role in conceptualising infectious illness transmission processes and successfully investigating illness dynamics for control strategies [6]. The most important components of the transmission phenomena of various illnesses may be identified through mathematical modeling. Esteva and Vargas developed the basic dengue fever modelling approach; they used a changing human population in their model and evaluated the system's stability [7, 8]. The influence of vaccination and antibody-dependent enhancement (ADE) in the phenomena of dengue fever has been hypothesized in [9, 10], while the scientists in [11, 12] organised the transmissions of dengue and tested the stability of equilibrium of the suggested system. Asymptomatic carriers of dengue disease are frequently reported and developed by scientists in [13, 14]; these carriers are most dangerous for noninfected areas of dengue infection. Dengue has a high rate of reinfection, making management of the disease more challenging. To better properly reflect dengue fever, researchers must look at the transmission procedure, including the effects of vaccine, reinfection, medication, and asymptomatic carriers. As a result, we have decided to model the dengue transmission phenomena in terms of asymptomatic cases, reinfection, vaccination, and therapy.

Fractional calculus enables the description of memory effects and genetic traits of varied materials; fractional calculus has been found to be more ideal in representing real situation than typical integer order calculus. Memory is an important component of vector-borne illnesses that affect both the host and mosquitoes [15, 16]. Fractional derivatives can efficiently manage the influence of memory in biological systems. In biology, economics, mathematics, physics, and other branches of study, many real-world issues are efficiently modelled in [17, 18]. In the research [19, 20], fractional operators have been used to simulate and explore the transmission dynamics of dengue illness. The fractional dynamics of dengue fever were examined using actual data and parameter estimates in [21]. Defterli [22] investigated the influence of temperature and conducted a comparative analysis of fractional-order models. A key component of vector-borne illnesses is the index of memory, which may be accurately expressed using a fractional structure. Therefore, fractional calculus is utilized to construct the transmission phenomena of dengue fever to emphasize the importance of memory in prevention of the infection.

The article "Qualitative Analysis of the Transmission Dynamics of Dengue with the Effect of Memory, Reinfection, and Vaccination" was published in 2022. Journal: Comput Math Methods Med.

The paper pattern is presented as follows: the rudimentary principle and findings of fractional theory are presented in Section 2. To depict a more realistic perspective of the transmission phenomena of dengue fever, we developed an epidemic model comprising vaccination, asymptotic fraction, reinfection, and therapy in Section 3.  Section 4 explores the proposed model, while Section 5 provides the Ulam-Hyers stability requirements. In Section 6, we provided a numerical technique for solving the suggested model and numerically examined the dengue dynamics as a function of various input factors of the system. In the last section, the article's conclusion and final remark are offered.

## 2. Theory of Fractional Calculus

We shall list the essential notions and terminology of fractional theory in this part, which will be used to analyse the hypothesized model. Memory is a key factor in the transmission phenomena of dengue infection which can be accurately represented through fractional-calculus. To be more specific, the researchers focused on fractional systems due to its wide applications. The rudimentary notions are given as follows.

**Definition 1 (see [23]).**

Assume *b*(*t*) be a function with the condition *b*(*t*) ∈ *L*^1^([*g*, *h*], *R*) and take the fractional order *ℏ*, then

(1) I ℏg+gbt=1Γℏ∫0tt−rℏ−1brdr

represents fractional integral and 0 < *ℏ* ≤ 1.

**Definition 2 (see [23]).**

Consider *b*(*t*) be a function with *b*(*t*) ∈ *C*^*n*^[*g*, *h*], then

(2) D LC0+ℏbt=1Γn−ℏ∫0tt−rn−ℏ−1hnrdr

represents the renowned derivative of Caputo.

**Lemma 1 (see [23]).**

Assume a function *b*(*h*) and take the below system

(3) D LC0+ℏbt=vt,t∈0,τ,n−1<ℏ<n,b0=v0,

where *v*(*t*) ∈ *C*([0, *τ*]), then

(4) $$\begin{array}{c} b\left(t\right)=\overset{n-1}{\underset{i=0}{\sum }}d_{i}t^{i},\text{for }i=0,1,\cdots ,n-1,\;d_{i}\in R. \end{array}$$

**Definition 3 (see [24]).**

The article "Qualitative Analysis of the Transmission Dynamics of Dengue with the Effect of Memory, Reinfection, and Vaccination" was published in 2022. Journal: Comput Math Methods Med.

The following is the Laplace transform for the Caputo operator.

(5) $$\begin{array}{c} £\left[{\;}^{LC}D_{0^{+}}^{\hbar }b\left(t\right)\right]=r^{\hbar }b\left(r\right)-\overset{n-1}{\underset{k=0}{\sum }}r^{\hbar -k-1}b^{k}\left(0\right), \end{array}$$

with *n* − 1 < *ℏ* < *n*. In addition to this, take the norm on *𝒳* as

(6) $$\begin{array}{c} \left\|b\right\|=\underset{t\in \left[0,\tau \right]}{\max}\left\{\left|b\right|,\text{for all }b\in X\right\}. \end{array}$$

**Theorem 1 (see [25]).**

Assume *𝒳* to be a Banach space in a way that *G* : *𝒳*⟶*𝒳* is compact and continuous. Then, one can find a fixed point of *G*, if

(7) $$\begin{array}{c} E=\left\{b\in X:b=\lambda Gb,\lambda \in \left(0,1\right)\right\} \end{array}$$

is bounded.

## 3. Formulation of Dengue Dynamics

In this formulation, we construct the interactions of female vectors *N*_*v*_ and hosts *N*_*h*_ to indicate the transmission process of dengue fever. The vector size is categorized into (*S*_*v*_) susceptible, (*E*_*v*_) susceptible, and (*I*_*v*_) infected compartments while the host population is divided into (*S*_*h*1_) susceptible, (*S*_*h*2_) susceptible after losing immunity, (*E*_*h*_) exposed, (*I*_*h*_) infected, (*I*_*hA*_) asymptomatic, and (*R*_*h*_) recovered compartments. We indicated the rate of transmission from *S*_*v*_ to *E*_*v*_ by ((*bβ*_*v*_/*N*_*h*_)(*I*_*h*_ + *I*_*hA*_)) while the rate of transmission from susceptible (*S*_*h*1_) and susceptible (*S*_*h*2_) to *E*_*v*_ are represented by *bβ*_*h*1_/*N*_*h*_*I*_*v*_ and (*bβ*_*h*2_/*N*_*h*_)*I*_*v*_. In addition to this, the transfer rate from *E*_*h*_ and *I*_*v*_ is symbolised by *ρ*_*h*_ and *ρ*_*v*_. The natural birth and mortality rates were assumed to remain constant for both populations, which are denoted by *μ*_*v*_ and *μ*_*h*_ for vector and host, accordingly.

A portion *ψ* is assumed to be asymptomatic, and recovery term is specified by *γ* from the infected classes. The terms *τ* and *p* represent the treatment and vaccination rates, whereas *b* represents the vector bite rate. Furthermore, a term *ν* of the *R*_*h*_ class loses immunity and becomes *S*_*h*2_ with a lower transmission rate *β*_*h*2_, resulting in *β*_*h*2_ < *β*_*h*1_. Then, we have below dynamics of dengue

(8) $$\begin{array}{c} \left\{\begin{array}{c} {\;}_{0}^{LC}D_{t}^{\vartheta }S_{h_{1}}=\mu_{h}^{\vartheta }N_{h}-\frac{\beta_{h1}b^{\vartheta }}{N_{h}}S_{h1}I_{v}-p^{\vartheta }S_{h1}-\mu_{h}^{\vartheta }S_{h1},\\ {\;}_{0}^{LC}D_{t}^{\vartheta }S_{h2}=\nu^{\vartheta }R_{h}-\frac{\beta_{h2}b^{\vartheta }}{N_{h}}S_{h2}I_{v}-\mu_{h}^{\vartheta }S_{h2},\\ \begin{array}{c} {\;}_{0}^{LC}D_{t}^{\vartheta }E_{h}=\frac{\beta_{h1}b^{\vartheta }}{N_{h}}S_{h1}I_{v}+\frac{\beta_{h2}b^{\vartheta }}{N_{h}}S_{h2}I_{v}-\left(\rho_{h}^{\vartheta }+\mu_{h}^{\vartheta }\right)E_{h},\\ {\;}_{0}^{LC}D_{t}^{\vartheta }I_{h}=\left(1-\psi \right)\rho_{h}^{\vartheta }E_{h}-\left(\tau^{\vartheta }+\gamma^{\vartheta }+\mu_{h}^{\vartheta }\right)I_{h},\\ \begin{array}{c} {\;}_{0}^{LC}D_{t}^{\vartheta }I_{hA}=\psi \rho_{h}^{\vartheta }E_{h}-\left(\gamma^{\vartheta }+\mu_{h}^{\vartheta }\right)I_{hA},\\ {\;}_{0}^{LC}D_{t}^{\vartheta }R_{h}=p^{\vartheta }S_{h1}+\tau^{\vartheta }I_{h}+\gamma^{\vartheta }\left(I_{h}+I_{hA}\right)-\left(\mu_{h}^{\vartheta }+\nu^{\vartheta }\right)R_{h},\\ \begin{array}{c} {\;}_{0}^{LC}D_{t}^{\vartheta }S_{v}=\mu_{v}^{\vartheta }N_{v}-\frac{\beta_{v}b^{\vartheta }}{N_{h}}\left(I_{h}+I_{hA}\right)S_{v}-\mu_{v}^{\vartheta }S_{v},\\ {\;}_{0}^{LC}D_{t}^{\vartheta }E_{v}=\frac{\beta_{v}b^{\vartheta }}{N_{h}}\left(I_{h}+I_{hA}\right)S_{v}-\left(\rho_{v}^{\vartheta }+\mu_{v}^{\vartheta }\right)E_{v},\\ {\;}_{0}^{LC}D_{t}^{\vartheta }I_{v}=\rho_{v}^{\vartheta }E_{v}-\mu_{v}^{\vartheta }I_{v}, \end{array} \end{array} \end{array} \end{array}\right. \end{array}$$

where

(9) $$\begin{array}{c} S_{v}\left(0\right)\geq 0,\\ E_{v}\left(0\right)\geq 0,\\ I_{v}\left(0\right)\geq 0,\\ S_{h1}\left(0\right)\geq 0,\\ S_{h2}\left(0\right)\geq 0,\\ E_{h}\left(0\right)\geq 0,\\ I_{h}\left(0\right)\geq 0,\\ I_{hA}\left(0\right)\geq 0,\\ R_{h}\left(0\right)\geq 0. \end{array}$$

Furthermore, the strength of species is

(10) $$\begin{array}{c} N_{v}=S_{v}+E_{v}+I_{v},\\ N_{h}=S_{h1}+S_{h2}+E_{v}+I_{h}+I_{hA}+R_{h}. \end{array}$$

Liouville-Caputo's operator is denoted by  _0_^*LC*^*D*_*t*_^*ϑ*^, while the memory index is denoted by *ϑ*. Because biological processes are nonlocal, the outcomes of fractional systems are more dependable and precise; also, fractional systems contain hereditary properties and convey knowledge about their past and present states for the future. Because it is commonly known that Caputo's derivative is more trustworthy and versatile for analysis, we used a fractional framework to depict the dynamics of dengue disease.

The article "Qualitative Analysis of the Transmission Dynamics of Dengue with the Effect of Memory, Reinfection, and Vaccination" was published in 2022. Journal: Comput Math Methods Med.

**Theorem 2 .**

The solutions (*S*_*h*1_, *S*_*h*2_, *E*_*h*_, *I*_*h*_, *I*_*hA*_, *R*_*h*_, *S*_*v*_, *E*_*v*_, *I*_*v*_) of the fractional model (8) of dengue infection are positive and bounded.

**Proof**

In order to obtain the required result, we proceed as follows:

(11) D0LCtϑSh1Sh1=0=μhϑNh≥0,D0LCtϑSh2Sh2=0νϑRh≥0,D0LCtϑEhEh=0=βh1bϑNhSh1Iv+βh2bϑNhSh2Iv≥0,D0LCtϑIhIh=0=ρhϑ1−ψEh≥0,D0LCtϑIhAIhA=0=ρhϑψEh≥0,D0LCtϑRhRh=0=pϑSh1+γϑIh+IhA+τϑIh≥0,D0LCtϑSvSv=0=μvϑNv≥0,D0LCtϑEvEv=0=βvbϑNhIh+IhASv≥0,D0LCtϑIvIv=0=ρvϑEv≥0.

Hence, our fractional system (8) is positive. To show that the solution is bounded, we first add all the compartments of host population as

(12) $$\begin{array}{c} {}_{0}^{LC}D_{t}^{\vartheta }\left(S_{h1}+S_{h2}+E_{h}+I_{h}+I_{hA}+R_{h}\right)\leq M-\mu_{h}^{\vartheta }\left(S_{h1}+S_{h2}+E_{h}+I_{h}+I_{hA}+R_{h}\right), \end{array}$$

where *ℳ* = *μ*_*h*_^*ϑ*^*N*_*h*_. We obtained the following by solving the above:

(13) $$\begin{array}{c} \left(S_{h1}+S_{h2}+E_{h}+I_{h}+I_{hA}+R_{h}\right)\leq \left(S_{h1}\left(0\right)+S_{h2}\left(0\right)+E_{h}\left(0\right)+I_{h}\left(0\right)+I_{hA}\left(0\right)+R_{h}\left(0\right)-\frac{M}{\mu_{h}^{\vartheta }}\right)E_{\vartheta }\left(-\mu_{h}^{\vartheta }t^{\vartheta }\right)+\frac{M}{\mu_{h}^{\vartheta }}. \end{array}$$

We get the following by asymptotic behavior of Mittag-Leffler function [23]:

(14) $$\begin{array}{c} \left(S_{h1}+S_{h2}+E_{h}+I_{h}+I_{hA}+R_{h}\right)\leq \frac{M}{\mu_{h}^{\vartheta }}≅M_{1}. \end{array}$$

In the same way, we can take the compartments of vector population of the system (8); we have *S*_*v*_ + *E*_*v*_ + *I*_*v*_ ≤ *ℳ*_2_, in which *ℳ*_2_ = *𝒩*/*μ*_*v*_^*ϑ*^. Consequently, the solution of the system (8) is positive and bounded.

Our suggested fractional model (8) of dengue infection's disease-free stable state is represented by *ℰ*_0_(*S*_*h*1_, *S*_*h*2_, *E*_*h*_, *I*_*h*_, *I*_*hA*_, *R*_*h*_, *S*_*v*_, *E*_*v*_, *I*_*v*_) and is provided by

(15) $$\begin{array}{c} E_{0}=\left(L_{1},L_{2},0,0,0,L_{3},N_{v}^{0},0,0\right), \end{array}$$

where *ℒ*_1_ = *μ*_*h*_^*ϑ*^*N*_*h*_^0^/*p*^*ϑ*^ + *μ*_*h*_^*ϑ*^, *ℒ*_2_ = *ν*_*h*_^*ϑ*^*p*^*ϑ*^/(*p*^*ϑ*^ + *μ*_*h*_^*ϑ*^)(*ν*^*ϑ*^ + *μ*_*h*_^*ϑ*^), and *ℒ*_3_ = *μ*_*h*_^*ϑ*^*p*^*ϑ*^*N*_*h*_^0^/(*p*^*ϑ*^ + *μ*_*h*_^*ϑ*^)(*ν*^*ϑ*^ + *μ*_*h*_^*ϑ*^). In this study, we mainly focused on the dynamical behavior and qualitative analysis of the infection; however, stability, sensitivity, bifurcation, and optimal control will be explored in our future work.

## 4. Theory of Existence

The qualitative character of the suggested fractional model (8) of dengue disease will be examined in this phase of the study using existence theory. To accomplish so, we must follow the instructions outlined below:

(16) $$\begin{array}{c} \left\{\begin{array}{c} P_{1}\left(t,S_{h1},S_{h2},E_{h},I_{h},I_{hA},S_{v},E_{v},I_{v}\right)=\mu_{h}^{\vartheta }N_{h}-\frac{\beta_{h1}b^{\vartheta }}{N_{h}}S_{h1}I_{v}-p^{\vartheta }S_{h1}-\mu_{h}^{\vartheta }S_{h1},\\ P_{2}\left(t,S_{h1},S_{h2},E_{h},I_{h},I_{hA},S_{v},E_{v},I_{v}\right)=\nu^{\vartheta }R_{h}-\frac{\beta_{h2}b^{\vartheta }}{N_{h}}S_{h2}I_{v}-\mu_{h}^{\vartheta }S_{h2},\\ P_{3}\left(t,S_{h1},S_{h2},E_{h},I_{h},I_{hA},S_{v},E_{v},I_{v}\right)=\frac{\beta_{h1}b^{\vartheta }}{N_{h}}S_{h1}I_{v}+\frac{\beta_{h2}b^{\vartheta }}{N_{h}}S_{h2}I_{v}-\left(\mu_{h}^{\vartheta }+\rho_{h}^{\vartheta }\right)E_{h},\\ P_{4}\left(t,S_{h1},S_{h2},E_{h},I_{h},I_{hA},S_{v},E_{v},I_{v}\right)=\left(1-\psi \right)\rho_{h}^{\vartheta }E_{h}-\left(\gamma^{\vartheta }+\mu_{h}^{\vartheta }+\tau^{\vartheta }\right)I_{h},\\ P_{5}\left(t,S_{h1},S_{h2},E_{h},I_{h},I_{hA},S_{v},E_{v},I_{v}\right)=\psi \rho_{h}^{\vartheta }E_{h}-\left(\gamma^{\vartheta }+\mu_{h}^{\vartheta }\right)I_{hA},\\ P_{6}\left(t,S_{h1},S_{h2},E_{h},I_{h},I_{hA},S_{v},E_{v},I_{v}\right)=p^{\vartheta }S_{h1}+\tau^{\vartheta }I_{h}+\gamma^{\vartheta }\left(I_{h}+I_{hA}\right)-\left(\mu_{h}^{\vartheta }+\nu^{\vartheta }\right)R_{h},\\ P_{7}\left(t,S_{h1},S_{h2},E_{h},I_{h},I_{hA},S_{v},E_{v},I_{v}\right)=\mu_{v}^{\vartheta }N_{v}-S_{v}\frac{b^{\vartheta }\beta_{v}}{N_{h}}\left(I_{h}+I_{hA}\right)-\mu_{v}^{\vartheta }S_{v},\\ P_{8}\left(t,S_{h1},S_{h2},E_{h},I_{h},I_{hA},S_{v},E_{v},I_{v}\right)=\frac{b^{\vartheta }\beta_{v}}{N_{h}}S_{v}\left(I_{h}+I_{hA}\right)-\left(\mu_{v}^{\vartheta }+\rho_{v}^{\vartheta }\right)E_{v},\\ P_{9}\left(t,S_{h1},S_{h2},E_{h},I_{h},I_{hA},S_{v},E_{v},I_{v}\right)=\rho_{v}^{\vartheta }E_{v}-\mu_{v}^{\vartheta }I_{v}. \end{array}\right. \end{array}$$

We can also rewrite the system (16) as

(17) $$\begin{array}{c} \left\{\begin{array}{cc} {}^{LC}D_{0^{+}}^{\vartheta }P\left(t\right)=Z\left(t,P\left(t\right)\right), & t\in \left[0,\tau \right],\\ P\left(0\right)=P_{0}, & 0<\vartheta \leq 1, \end{array}\right. \end{array}$$

where

(18) $$\begin{array}{c} \left\{\begin{array}{cc} P\left(t\right)= & S_{h1}\left(t\right),\\ & S_{h2}\left(t\right),\\ & E_{h}\left(t\right),\\ & I_{h}\left(t\right),\\ & I_{hA}\left(t\right),\\ & R_{h}\left(t\right),\\ & S_{v}\left(t\right),\\ & E_{v}\left(t\right),\\ & I_{v}\left(t\right), \end{array}\right.\\ \left\{\begin{array}{cc} P_{0}\left(t\right)= & S_{h10},\\ & S_{h20},\\ & E_{h0},\\ & I_{h0},\\ & I_{hA0},\\ & R_{h0},\\ & S_{v0},\\ & E_{v0},\\ & I_{v0}, \end{array}\right.\\ \left\{\begin{array}{cc} Z\left(t,P\left(t\right)\right)= & P_{1}\left(t,S_{h1},S_{h2},E_{h},I_{h},I_{hA},R_{h},S_{v},E_{v},I_{v}\right),\\ & P_{2}\left(t,S_{h1},S_{h2},E_{h},I_{h},I_{hA},R_{h},S_{v},E_{v},I_{v}\right),\\ & P_{3}\left(t,S_{h1},S_{h2},E_{h},I_{h},I_{hA},R_{h},S_{v},E_{v},I_{v}\right),\\ & P_{4}\left(t,S_{h1},S_{h2},E_{h},I_{h},I_{hA},R_{h},S_{v},E_{v},I_{v}\right),\\ & P_{5}\left(t,S_{h1},S_{h2},E_{h},I_{h},I_{hA},R_{h},S_{v},E_{v},I_{v}\right),\\ & P_{6}\left(t,S_{h1},S_{h2},E_{h},I_{h},I_{hA},R_{h},S_{v},E_{v},I_{v}\right),\\ & P_{7}\left(t,S_{h1},S_{h2},E_{h},I_{h},I_{hA},R_{h},S_{v},E_{v},I_{v}\right),\\ & P_{8}\left(t,S_{h1},S_{h2},E_{h},I_{h},I_{hA},R_{h},S_{v},E_{v},I_{v}\right),\\ & P_{9}\left(t,S_{h1},S_{h2},E_{h},I_{h},I_{hA},R_{h},S_{v},E_{v},I_{v}\right). \end{array}\right. \end{array}$$

Through upper mentioned Lemma 3, the system (17) can be written in equivalent integral shape as given below:

(19) $$\begin{array}{c} P\left(t\right)=P_{0}\left(t\right)+\frac{1}{\Gamma \left(\vartheta \right)}\int_{0}^{t}{\left(t-r\right)}^{\vartheta -1}Z\left(r,P\left(r\right)\right)dr. \end{array}$$

For the examination of our suggested system, we use the Lipschitz criteria listed as follows:

C1. For *q* ∈ [0, 1), there exists *𝒰*_*𝒵*_, *𝒱*_*𝒵*_ with the following

(20) $$\begin{array}{c} \left|Z\left(t,P\left(t\right)\right)\right|\leq U_{P}{\left|P\right|}^{q}+V_{Z}. \end{array}$$

C2. We have *M*_*𝒵*_ > 0, and all *𝒫*, $\bar{𝒫}\in 𝒳$, with the condition

(21) $$\begin{array}{c} \left|Z\left(t,P\right)-Z\left(t,\bar{P}\right)\right|\leq M_{Z}\left[\left|P-\bar{P}\right|\right]. \end{array}$$

Introduce a map *B* on *𝒳* as given below:

(22) $$\begin{array}{c} BP\left(t\right)=P_{0}\left(t\right)+\frac{1}{\Gamma \left(\vartheta \right)}\int_{0}^{t}{\left(t-r\right)}^{\vartheta -1}Z\left(r,P\left(r\right)\right)dr. \end{array}$$

There is at least a solution of (17), if the C1 and C2 holds true. To investigate the solution of our dengue system, we proceed as follows.

The article "Qualitative Analysis of the Transmission Dynamics of Dengue with the Effect of Memory, Reinfection, and Vaccination" was published in 2022. Journal: Comput Math Methods Med.

**Theorem 3 .**

There exists at least one solution of the suggested model (8) of dengue fever if the assumptions C1 and C2 satisfied.

**Proof**

We will utilize Schaefer's fixed point theorem to show the needed result. We will demonstrate this theorem in four phases, as follows:

P1. In first phase, the continuity of the operator *B* will be established. Take here, *𝒫*_*i*_ is continuous for *i* = 1, 2, ⋯, 9; this gives us that *𝒵*(*t*, *𝒫*(*t*)) is continuous. In the upcoming steps, *𝒫*_*j*_, *𝒫* ∈ *𝒳* such that *𝒫*_*j*_⟶*𝒫*, we have *B𝒫j*⟶*B𝒫*. In addition to this, assume

(23) $$\begin{array}{c} \left\|BP_{j}-BP\right\|=\underset{t\in \left[0,\tau \right]}{\max}\left|\frac{1}{\Gamma \left(\vartheta \right)}\int_{0}^{t}{\left(t-r\right)}^{\vartheta -1}Q_{j}\left(r,P_{j}\left(r\right)\right)dr-\frac{1}{\Gamma \left(\vartheta \right)}\int_{0}^{t}{\left(t-r\right)}^{\vartheta -1}Z\left(r,P\left(r\right)\right)ds\right|\leq \underset{t\in \left[0,\tau \right]}{\max}\int_{0}^{t}\left|\frac{{\left(t-r\right)}^{\vartheta -1}}{\Gamma \left(\vartheta \right)}\right|\left|Z_{j}\left(r,P_{j}\left(r\right)\right)-Z\left(r,P\left(r\right)\right)\right|dr\leq \frac{\tau^{\vartheta }M_{Z}}{\Gamma \left(\vartheta +1\right)}\left\|P_{j}-P\right\|⟶0\text{ as }j⟶\infty . \end{array}$$

The continuity of *B𝒫j*⟶*B𝒫* is achieved as *𝒵* is continuous which insure the continuity of *B*.

The article "Qualitative Analysis of the Transmission Dynamics of Dengue with the Effect of Memory, Reinfection, and Vaccination" was published in 2022. Journal: Comput Math Methods Med.

P2. In the second phase, the boundedness of *B* will be established. Let us take *𝒫* ∈ X, then the following are satisfied through the operator *B*:

(24) $$\begin{array}{c} \left\|BP\right\|=\underset{t\in \left[0,\tau \right]}{\max}\left|P_{o}\left(t\right)+\frac{1}{\Gamma \left(\vartheta \right)}\int_{0}^{t}{\left(t-r\right)}^{\vartheta -1}Z\left(r,P\left(r\right)\right)dr\right|\leq \left|P_{0}\right|\underset{t\in \left[0,\tau \right]}{\max}\frac{1}{\Gamma \left(\vartheta \right)}\int_{0}^{t}\left|{\left(t-r\right)}^{\vartheta -1}\right|\left|Z\left(r,P\left(r\right)\right)\right|dr\leq \left|P_{0}\right|+\frac{\tau^{\vartheta }}{\Gamma \left(\vartheta +1\right)}\left\{U_{Z}{\left\|P\right\|}^{q}+V_{Z}\right\}. \end{array}$$

Next, the boundedness of *B*(*T*) will be established for a bounded subset *T* of *𝒳*. Assume *𝒫* ∈ *T* as *S* is bounded; as a result of this, there is a *U* ≥ 0 such that

(25) $$\begin{array}{c} \left\|P\right\|\leq U,\forall P\in T. \end{array}$$

As a result, we get the following through the above for any *𝒫* ∈ *T*:

(26) $$\begin{array}{c} \left\|BW\right\|\leq \left|P_{0}\right|+\frac{\tau^{\vartheta }}{\Gamma \left(\vartheta +1\right)}\left[U_{Z}{\left\|P\right\|}^{q}+V_{Z}\right]\leq \left|P_{0}\right|+\frac{\tau^{\vartheta }}{\Gamma \left(\vartheta +1\right)}\left[U_{Z}U^{q}+V_{Z}\right]. \end{array}$$

Consequently, the boundedness of the operator *B*(*T*) is obtained.

P3. For the equi-continuity, take *t*_1_, *t*_2_ ∈ [0, *τ*] with *t*_1_ ≥ *t*_2_, then we have

(27) $$\begin{array}{c} \left|BP\left(t_{1}\right)-BP\left(t_{1}\right)\right|=\left|\frac{1}{\Gamma \left(\vartheta \right)}\int_{0}^{t_{1}}\left|{\left(t_{1}-r\right)}^{\vartheta -1}\right|\left|Z\left(r,P\left(r\right)\right)\right|dr-\frac{1}{\Gamma \left(\vartheta \right)}\int_{0}^{t_{2}}\left|{\left(t_{2}-r\right)}^{\vartheta -1}\right|\left|Z\left(r,P\left(r\right)\right)\right|dr\right|\leq \left|\frac{1}{\Gamma \left(\vartheta \right)}\int_{0}^{t_{1}}\left|{\left(t_{1}-r\right)}^{\vartheta -1}\right|-\frac{1}{\Gamma \left(\vartheta \right)}\int_{0}^{t_{2}}\left|{\left(t_{2}-r\right)}^{\vartheta -1}\right|\right|\left|Z\left(r,P\left(r\right)\right)\right|dr\leq \frac{\tau^{\vartheta }}{\Gamma \left(\vartheta +1\right)}\left[U_{Z}{\left\|P\right\|}^{q}+V_{Z}\right]\left[t_{1}^{\vartheta }-t_{2}^{\vartheta }\right], \end{array}$$

which goes to zero as *t*_1_ goes to *t*_2_. This insures the relative compactness of *B*(*T*) through Arzela-Ascoli theorem.

The article "Qualitative Analysis of the Transmission Dynamics of Dengue with the Effect of Memory, Reinfection, and Vaccination" was published in 2022. Journal: Comput Math Methods Med.

P4. In fourth phase, the following set is considered:

(28) $$\begin{array}{c} E=\left\{P\in X:P=\lambda BP,\lambda \in \left(0,1\right)\right\}. \end{array}$$

To show that set *ℰ* is bounded, we assume *𝒫* ∈ *ℰ*; then for any *t* ∈ [0, *τ*], the below condition satisfies

(29) $$\begin{array}{c} \left\|P\right\|=\lambda \left\|BP\right\|\leq \lambda \left[\left|P_{0}\right|\frac{\tau^{\vartheta }}{\Gamma \left(\vartheta +1\right)}\left[U_{Z}{\left\|P\right\|}^{q}+V_{Z}\right]\right]. \end{array}$$

This indicates that the set *ℰ* is bounded. As a result of Schaefer's theorem, the operator *B* has a fixed point. Consequently, our suggested system (17) of dengue has at least one solution.

**Remark 1 .**

If C1 fulfills for *q* = 1, then Theorem 7 can be proved for (*τ*^*ϑ*^*U*_*Z*_/Γ(*ϑ* + 1)) < 1.

**Theorem 4 .**

If (*τ*^*ϑ*^*U*_*Z*_/Γ(*ϑ* + 1)) < 1 is satisfied, then the dengue fever fractional system (17) has a unique solution.

**Proof**

For the proof, Banach's contraction theorem is applied with the assumption $𝒫,\bar{𝒫}\in 𝒳$ as

(30) $$\begin{array}{c} \left\|BP-B\bar{P}\right\|\leq \underset{x⟶\infty }{\max}\frac{1}{\Gamma \left(\vartheta \right)}\int_{0}^{t}\left|{\left(t-r\right)}^{\vartheta -1}\right|\left|Z\left(r,P\left(r\right)\right)-Z\left(r,\bar{P}\left(r\right)\right)\right|dr\leq \frac{\tau^{\vartheta }U_{Z}}{\Gamma \left(\vartheta +1\right)}\left\|P-\bar{P}\right\|. \end{array}$$

Thus, there is a unique fixed point of *B*; therefore, a unique of model (17) of dengue fever exists.

## 5. Ulam-Hyers Stability

Here, our main focus is to investigate the suggested model of dengue for the Ulam-Hyers stability (UHS). First, Ullam proposed the concept of stability in 1940, and Hyers [26, 27] expanded it. Several researchers have applied the Ulam-Hyers stability concept to several fields of study [28–30]. The fundamental theory is as follows.

Let us consider *𝒦* : *𝒳*⟶*𝒳* in a way that

(31) $$\begin{array}{c} KV=V\text{ for }V\in X. \end{array}$$

**Definition 4 .**

Upper mentioned (31) is UHS if for every solution *𝒫* ∈ *𝒳* and *ζ* > 0, one can find

(32) $$\begin{array}{c} \left\|V-KV\right\|\leq \zeta \text{ for }t\in \left[0,\tau \right]. \end{array}$$

Furthermore, there exists a unique solution $\bar{𝒫}$ of the upper mentioned (31) in a way that 0 < *𝒞*_*q*_ and the following holds true

(33) $$\begin{array}{c} \left\|\bar{V}-V\right\|\leq C_{q}\zeta ,\;t\in \left[0,\tau \right]. \end{array}$$

**Definition 5 .**

Let *𝒫* and $\bar{𝒫}$ be solution of (31); then, the system (31) is generalized UHS if

(34) $$\begin{array}{c} \left\|\bar{V}-V\right\|\leq Z\left(\zeta \right), \end{array}$$

in which the image of 0 is 0 and *𝒵* ∈ *C*(*R*, *R*).

The article "Qualitative Analysis of the Transmission Dynamics of Dengue with the Effect of Memory, Reinfection, and Vaccination" was published in 2022. Journal: Comput Math Methods Med.

**Remark 2 .**

If the solution $\bar{𝒫}\in 𝒳$ satisfies (33) and for all *t* ∈ [0, *τ*] the below satisfied

- |*ϖ*(*t*)| ≤ *ζ*, in which *ϖ* ∈ *C*([0, *τ*]; *R*)
- $𝒦\bar{𝒱}\left(T\right)=\bar{𝒱}+\varpi \left(T\right)$

Then, system (17) after small changes becomes as

(35) D C0+ϑVt=Pt,Vt+ϖt,V0=V0.

**Lemma 2 .**

System (35) also fulfills

(36) $$\begin{array}{c} \left|V\left(t\right)-TV\left(t\right)\right|\leq a\zeta ,\;\text{in which }a=\frac{\tau^{\vartheta }}{\Gamma \left(\vartheta +1\right)}. \end{array}$$

Utilizing Lemma 3 and Remark 12, we can easily prove this theorem.

**Theorem 5 .**

If the condition (*τ*^*ϑ*^*L*_*𝒫*_/Γ(*ϑ* + 1)) < 1 holds true, then the solution of (17) is UHS and generalized UHS on Lemma 13.

**Proof**

We assume the solutions *𝒱* ∈ *X* and $\bar{𝒱}\in X$ of the system (17) for the required proof, thus

(37) $$\begin{array}{c} \left|V\left(t\right)-\bar{V}\left(t\right)\right|=\left|V\left(t\right)-\bar{V}\left(t\right)\right|\leq \left|V\left(t\right)-T\bar{V}\left(t\right)\right|\leq \left|V\left(t\right)-T\bar{V}\left(t\right)\right|\leq a\zeta +\frac{\tau^{\xi }L_{U}}{\Gamma \left(\xi +1\right)}\left|V\left(t\right)-\bar{V}\left(t\right)\right|\leq \frac{a\zeta }{1-\left(\tau^{\xi }L_{U}/\Gamma \left(\xi +1\right)\right)}. \end{array}$$

Thus, the UHS and GUHS of the suggested noninteger system (17) of dengue fever are insured.

**Definition 6 .**

The solution of (31) is the Ulam-Hyers-Rassias stable (UHRS) if for any *𝒱* ∈ *𝒳*, we write

(38) $$\begin{array}{c} \left\|V-KV\right\|\leq \Omega \left(t\right)\zeta ,\text{for }t\in \left[0,\tau \right], \end{array}$$

where *Ω* ∈ *C*[[0, *τ*], *R*] and *ζ* > 0. If *𝒞*_*q*_ > 0, then there exists a unique solution $\bar{𝒱}$ of the system (31) satisfying

(39) $$\begin{array}{c} \left\|\bar{V}-V\right\|\leq C_{q}\Omega \left(t\right)\zeta , \end{array}$$

for all *t* in [0, *τ*].

**Definition 7 .**

Take the unique solution $\bar{𝒫}$ and *𝒫* be any other solution of (31) such that

(40) $$\begin{array}{c} \left\|\bar{V}-V\right\|\leq C_{q,\Omega }\Omega \left(t\right)\zeta , \end{array}$$

in which *t* belongs to [0, *τ*], *Ω* ∈ *D*[[0, *τ*], *R*] in a way that *C*_*q*,*Ω*_ and *ζ* > 0. This implies that the solution of (31) is generalized UHRS.

**Remark 3 .**

Take $\bar{𝒱}\in X$; this solution will satisfy (33) if ∀*t* ∈ [0, *τ*], we write

- |*ϖ*(*t*)| ≤ *ζΩ*(*t*), in which *ϖ*(*t*) ∈ *𝒞*([0, *τ*]; *R*)
- $𝒦\bar{𝒱}\left(t\right)=\bar{𝒱}+\varpi \left(t\right)$

**Lemma 3 .**

The article "Qualitative Analysis of the Transmission Dynamics of Dengue with the Effect of Memory, Reinfection, and Vaccination" was published in 2022. Journal: Comput Math Methods Med.

The perturb system (17) holds the conditions

(41) $$\begin{array}{c} \left|V\left(t\right)-TV\left(T\right)\right|\leq a\Omega \left(t\right)\zeta ,\text{in which }a=\frac{\tau^{\vartheta }}{\Gamma \left(\vartheta +1\right)}. \end{array}$$

Utilizing Lemma 3 and Remark 17, we can easily obtained the required proof.

**Theorem 6 .**

The solution of (17) is UHRS and generalized UHRS on Lemma 18 if (*τ*^*ϑ*^*L*_*𝒰*_/Γ(*ϑ* + 1)) < 1 holds true.

**Proof**

Assuming a unique solution $\bar{𝒱}\in 𝒳$ and any other system (17) solution *𝒱* ∈ *𝒳*, we get that

(42) $$\begin{array}{c} \left|V\left(t\right)-\bar{V}\left(t\right)\right|=\left|V\left(t\right)-\bar{V}\left(t\right)\right|\leq \left|V\left(t\right)-T\bar{V}\left(t\right)\right|\leq \left|V\left(t\right)-T\bar{V}\left(t\right)\right|\leq a\Omega \left(t\right)\zeta +\frac{\tau^{\vartheta }L_{P}}{\Gamma \left(\vartheta +1\right)}\left|V\left(t\right)-\bar{V}\left(t\right)\right|\leq \frac{a\Omega \left(t\right)\zeta }{1-\left(\tau^{\vartheta }L_{P}/\Gamma \left(\vartheta +1\right)\right)}. \end{array}$$

As a result, UHRS and generalized UHRS are the solutions of (17).

## 6. Dynamical Behavior of the Model

Here, the dynamical behavior of the system of dengue infection will be investigated. The Laplace transform will be used to construct a scheme for the system (8). The method steps are given as

(43) $$\begin{array}{c} \left\{\begin{array}{c} L\left[S_{h1}\left(t\right)\right]=\frac{S_{h10}}{s}+\frac{1}{s^{\vartheta }}L\left[\mu_{h}^{\vartheta }N_{h}-\frac{\beta_{h1}b^{\vartheta }}{N_{h}}S_{h1}I_{v}-p^{\vartheta }S_{h1}-\mu_{h}^{\vartheta }S_{h1}\right],\\ L\left[S_{h2}\left(t\right)\right]=\frac{S_{h20}}{s}+\frac{1}{s^{\vartheta }}L\left[\nu^{\vartheta }R_{h}-\frac{\beta_{h2}b^{\vartheta }}{N_{h}}S_{h2}I_{v}-\mu_{h}^{\vartheta }S_{h2}\right],\\ L\left[E_{h}\left(t\right)\right]=\frac{E_{h0}}{s}+\frac{1}{s^{\vartheta }}L\left[\frac{\beta_{h1}b^{\vartheta }}{N_{h}}S_{h1}I_{v}+\frac{\beta_{h2}b^{\vartheta }}{N_{h}}S_{h2}I_{v}-\left(\mu_{h}^{\vartheta }+\rho_{h}^{\vartheta }\right)E_{h}\right],\\ L\left[I_{h}\left(t\right)\right]=\frac{I_{h0}}{s}+\frac{1}{s^{\vartheta }}L\left[\left(1-\psi \right)\rho_{h}^{\vartheta }E_{h}-\left(\tau^{\vartheta }+\gamma^{\vartheta }+\mu_{h}^{\vartheta }\right)I_{h}\right],\\ L\left[I_{hA}\left(t\right)\right]=\frac{I_{hA0}}{s}+\frac{1}{s^{\vartheta }}L\left[\psi \rho_{h}^{\vartheta }E_{h}-\left(\gamma^{\vartheta }+\mu_{h}^{\vartheta }\right)I_{hA}\right],\\ L\left[R_{h}\left(t\right)\right]=\frac{R_{h0}}{s}+\frac{1}{s^{\vartheta }}L\left[p^{\vartheta }S_{h1}+\tau^{\vartheta }I_{h}+\gamma^{\vartheta }\left(I_{h}+I_{hA}\right)-\left(\mu_{h}^{\vartheta }+\nu^{\vartheta }\right)R_{h}\right],\\ L\left[S_{v}\left(t\right)\right]=\frac{S_{v0}}{s}+\frac{1}{s^{\vartheta }}L\left[\mu_{v}^{\vartheta }N_{v}-\frac{b^{\vartheta }\beta_{v}}{N_{h}}S_{v}\left(I_{h}+I_{hA}\right)-\mu_{v}^{\vartheta }S_{v}\right],\\ L\left[E_{v}\left(t\right)\right]=\frac{E_{v0}}{s}+\frac{1}{s^{\vartheta }}L\left[\frac{b^{\vartheta }\beta_{v}}{N_{h}}S_{v}\left(I_{h}+I_{hA}\right)-\left(\mu_{v}^{\vartheta }+\rho_{v}^{\vartheta }\right)E_{v}\right],\\ L\left[I_{v}\left(t\right)\right]=\frac{I_{v0}}{s}+\frac{1}{s^{\vartheta }}L\left[\rho_{v}^{\vartheta }E_{v}-\mu_{v}^{\vartheta }I_{v}\right], \end{array}\right. \end{array}$$

where

(44) $$\begin{array}{c} \left\{\begin{array}{c} S_{h1}\left(t\right)=\overset{\infty }{\underset{j=0}{\sum }}S_{h1j}\left(t\right),S_{h2}\left(t\right)=\overset{\infty }{\underset{j=0}{\sum }}S_{h2j}\left(t\right),\\ E_{h}\left(t\right)=\overset{\infty }{\underset{j=0}{\sum }}E_{hj}\left(t\right),I_{h}\left(t\right)=\overset{\infty }{\underset{j=0}{\sum }}I_{hj}\left(t\right),\\ I_{hA}\left(t\right)=\overset{\infty }{\underset{j=0}{\sum }}I_{hAj}\left(t\right),R_{h}\left(t\right)=\overset{\infty }{\underset{j=0}{\sum }}R_{hj}\left(t\right),\\ S_{v}\left(t\right)=\overset{\infty }{\underset{j=0}{\sum }}S_{vj}\left(t\right),E_{v}\left(t\right)=\overset{\infty }{\underset{j=0}{\sum }}E_{vj}\left(t\right),\\ I_{v}\left(t\right)=\overset{\infty }{\underset{j=0}{\sum }}I_{vj}\left(t\right). \end{array}\right. \end{array}$$

We use Adomian polynomials to decompose the nonlinear terms as

(45) $$\begin{array}{c} S_{h1}\left(t\right)I_{v}\left(t\right)=\overset{\infty }{\underset{j=0}{\sum }}D_{j}\left(t\right),\;\text{with}\;D_{j}\left(t\right)=\frac{1}{j!}\frac{d^{j}}{dz^{j}}\left[\overset{j}{\underset{k=0}{\sum }}z^{k}S_{h1k}\left(t\right)\overset{j}{\underset{k=0}{\sum }}z^{k}I_{hk}\left(t\right)\right]z=0,\\ S_{h2}\left(t\right)I_{v}\left(t\right)=\overset{\infty }{\underset{j=0}{\sum }}E_{j}\left(t\right),\;\text{with}\;\;E_{j}\left(t\right)=\frac{1}{j!}\frac{d^{j}}{{dz}^{j}}\left[\overset{j}{\underset{k=0}{\sum }}z^{k}S_{h2k}\left(t\right)\overset{j}{\underset{k=0}{\sum }}z^{k}I_{vk}\left(t\right)\right]z=0,\\ S_{v}\left(t\right)\left(I_{h}\left(t\right)+I_{hA}\left(t\right)\right)=\overset{\infty }{\underset{j=0}{\sum }}F_{j}\left(t\right),\;\text{with}\;F_{j}\left(t\right)=\frac{1}{j!}\frac{d^{j}}{{dz}^{j}}\left[\overset{j}{\underset{k=0}{\sum }}z^{k}S_{vk}\left(t\right)\overset{j}{\underset{k=0}{\sum }}z^{k}\left(I_{hk}\left(t\right)+I_{hAk}\right)\right]z=0. \end{array}$$

Therefore, we get

(46) $$\begin{array}{c} \left\{\begin{array}{c} L\left[\overset{\infty }{\underset{j=0}{\sum }}S_{h1j}\left(t\right)\right]=\frac{S_{h10}}{s}+\frac{1}{s^{\alpha }}L\left[\mu_{h}^{\vartheta }N_{h}-\frac{\beta_{h1}b^{\vartheta }}{N_{h}}\overset{\infty }{\underset{j=0}{\sum }}D_{j}\left(t\right)-p^{\vartheta }\overset{\infty }{\underset{j=0}{\sum }}S_{h1j}\left(t\right)-\mu_{h}^{\vartheta }\overset{\infty }{\underset{j=0}{\sum }}S_{h1j}\left(t\right)\right],\\ L\left[\overset{\infty }{\underset{j=0}{\sum }}S_{h2j}\left(t\right)\right]=\frac{S_{h20}}{s}+\frac{1}{s^{\vartheta }}L\left[\nu^{\vartheta }\overset{\infty }{\underset{j=0}{\sum }}R_{hj}\left(t\right)-\frac{\beta_{h2}b^{\vartheta }}{N_{h}}\overset{\infty }{\underset{j=0}{\sum }}E_{j}\left(t\right)-\mu_{h}^{\vartheta }\overset{\infty }{\underset{j=0}{\sum }}S_{h2j}\left(t\right)\right],\\ L\left[\overset{\infty }{\underset{j=0}{\sum }}E_{hj}\left(t\right)\right]=\frac{E_{h0}}{s}+\frac{1}{s^{\vartheta }}L\left[\frac{\beta_{h1}b^{\vartheta }}{N_{h}}\overset{\infty }{\underset{j=0}{\sum }}D_{j}\left(t\right)+\frac{\beta_{h2}b^{\vartheta }}{N_{h}}\overset{\infty }{\underset{j=0}{\sum }}E_{j}\left(t\right)-\left(\mu_{h}^{\vartheta }+\rho_{h}^{\vartheta }\right)\overset{\infty }{\underset{j=0}{\sum }}E_{hj}\left(t\right)\right],\\ L\left[\overset{\infty }{\underset{j=0}{\sum }}I_{hj}\left(t\right)\right]=\frac{I_{h0}}{s}+\frac{1}{s^{\vartheta }}L\left[\rho_{h}^{\vartheta }\left(1-\psi \right)\overset{\infty }{\underset{j=0}{\sum }}E_{hj}\left(t\right)-\left(\gamma^{\vartheta }+\mu_{h}^{\vartheta }+\tau^{\vartheta }\right)\overset{\infty }{\underset{j=0}{\sum }}I_{hj}\left(t\right)\right],\\ L\left[\overset{\infty }{\underset{j=0}{\sum }}I_{hAj}\left(t\right)\right]=\frac{I_{hA0}}{s}+\frac{1}{s^{\vartheta }}L\left[\rho_{h}^{\vartheta }\psi \overset{\infty }{\underset{j=0}{\sum }}E_{hj}\left(t\right)-\left(\gamma^{\vartheta }+\mu_{h}^{\vartheta }\right)\overset{\infty }{\underset{j=0}{\sum }}I_{hAj}\left(t\right)\right],\\ L\left[\overset{\infty }{\underset{j=0}{\sum }}R_{hj}\left(t\right)\right]=\frac{R_{h0}}{s}+\frac{1}{s^{\vartheta }}L\left[p^{\vartheta }\overset{\infty }{\underset{j=0}{\sum }}S_{h1j}\left(t\right)+\gamma^{\vartheta }\overset{\infty }{\underset{j=0}{\sum }}\left(I_{hj}\left(t\right)+I_{hAj}\left(t\right)\right)+\tau^{\vartheta }I_{h}-\left(\nu^{\vartheta }+\mu_{h}^{\vartheta }\right)\overset{\infty }{\underset{j=0}{\sum }}R_{hj}\left(t\right)\right],\\ L\left[\overset{\infty }{\underset{j=0}{\sum }}S_{vj}\left(t\right)\right]=\frac{S_{v0}}{s}+\frac{1}{s^{\vartheta }}L\left[\mu_{v}^{\vartheta }N_{v}-\frac{\beta_{v}b^{\vartheta }}{N_{h}}\overset{\infty }{\underset{j=0}{\sum }}F_{j}\left(t\right)-\mu_{v}^{\vartheta }\overset{\infty }{\underset{j=0}{\sum }}S_{vj}\left(t\right)\right],\\ L\left[\overset{\infty }{\underset{j=0}{\sum }}E_{vj}\left(t\right)\right]=\frac{E_{v0}}{s}+\frac{1}{s^{\vartheta }}L\left[\frac{\beta_{v}b^{\vartheta }}{N_{h}}\overset{\infty }{\underset{j=0}{\sum }}F_{j}\left(t\right)-\left(\rho_{v}^{\vartheta }+\mu_{v}^{\vartheta }\right)\overset{\infty }{\underset{j=0}{\sum }}E_{vj}\left(t\right)\right],\\ L\left[\overset{\infty }{\underset{j=0}{\sum }}I_{vj}\left(t\right)\right]=\frac{I_{v0}}{s}+\frac{1}{s^{\vartheta }}L\left[\rho_{v}^{\vartheta }\overset{\infty }{\underset{j=0}{\sum }}E_{vj}\left(t\right)-\mu_{v}^{\vartheta }\overset{\infty }{\underset{j=0}{\sum }}I_{vj}\left(t\right)\right], \end{array}\right.\\ \left\{\begin{array}{c} L\left[S_{h10}\left(t\right)\right]=\frac{S_{h10}}{s},\\ L\left[S_{h20}\left(t\right)\right]=\frac{S_{h20}}{s},\\ L\left[E_{h0}\left(t\right)\right]=\frac{E_{h0}}{s},\\ L\left[I_{h0}\left(t\right)\right]=\frac{I_{h0}}{s},\\ L\left[I_{hA0}\left(t\right)\right]=\frac{I_{hA0}}{s},\\ L\left[R_{h0}\left(t\right)\right]=\frac{R_{h0}}{s},\\ L\left[S_{v0}\left(t\right)\right]=\frac{S_{v0}}{s},\\ L\left[E_{v0}\left(t\right)\right]=\frac{E_{v0}}{s},\\ L\left[I_{v0}\left(t\right)\right]=\frac{I_{v0}}{s}. \end{array}\right. \end{array}$$

Thus, we have

(47) $$\begin{array}{c} \left\{\begin{array}{c} L\left[S_{h11}\left(t\right)\right]=\frac{1}{s^{\vartheta }}L\left[\mu_{h}^{\vartheta }N_{h}-\frac{b^{\vartheta }\beta_{h1}}{N_{h}}D_{0}\left(t\right)-p^{\vartheta }S_{h10}\left(t\right)-\mu_{h}^{\vartheta }S_{h10}\left(t\right)\right],\\ L\left[S_{h21}\left(t\right)\right]=\frac{1}{s^{\vartheta }}L\left[\nu^{\vartheta }R_{h0}\left(t\right)-\frac{b^{\vartheta }\beta_{h2}}{N_{h}}E_{0}\left(t\right)-\mu_{h}^{\vartheta }S_{h20}\left(t\right)\right],\\ L\left[E_{h1}\left(t\right)\right]=\frac{1}{s^{\vartheta }}L\left[\frac{\beta_{h1}b^{\vartheta }}{N_{h}}D_{0}\left(t\right)+\frac{\beta_{h2}b^{\vartheta }}{N_{h}}E_{0}\left(t\right)-\left(\rho_{h}^{\vartheta }+\mu_{h}^{\vartheta }\right)E_{h0}\left(t\right)\right],\\ L\left[I_{h1}\left(t\right)\right]=\frac{1}{s^{\vartheta }}L\left[\left(1-\psi \right)\rho_{h}^{\vartheta }E_{h0}\left(t\right)-\left(\gamma^{\vartheta }+\tau^{\vartheta }++\mu_{h}^{\vartheta }\right)I_{h0}\left(t\right)\right],\\ L\left[I_{hA1}\left(t\right)\right]=\frac{1}{s^{\vartheta }}L\left[\psi \rho_{h}^{\vartheta }E_{h0}\left(t\right)-\left(\gamma^{\vartheta }+\mu_{h}^{\vartheta }\right)I_{hA0}\left(t\right)\right],\\ L\left[R_{h1}\left(t\right)\right]=\frac{1}{s^{\vartheta }}L\left[p^{\vartheta }S_{h10}\left(t\right)+\tau^{\vartheta }I_{h0}\left(t\right)+\gamma^{\vartheta }\left(I_{h0}\left(t\right)+I_{hA0}\left(t\right)\right)-\left(\mu_{h}^{\vartheta }+\nu^{\vartheta }\right)R_{h0}\left(t\right)\right],\\ L\left[S_{v1}\left(t\right)\right]=\frac{1}{s^{\vartheta }}L\left[\mu_{v}^{\vartheta }N_{v}-\frac{b^{\vartheta }\beta_{v}}{N_{h}}F_{0}\left(t\right)-\mu_{v}^{\vartheta }S_{v0}\left(t\right)\right],\\ L\left[E_{v1}\left(t\right)\right]=\frac{1}{s^{\vartheta }}L\left[\frac{b^{\vartheta }\beta_{v}}{N_{h}}F_{0}\left(t\right)-\left(\mu_{v}^{\vartheta }+\rho_{v}^{\vartheta }\right)E_{v0}\left(t\right)\right],\\ L\left[I_{v1}\left(t\right)\right]=\frac{1}{s^{\vartheta }}L\left[\rho_{v}^{\vartheta }E_{v0}\left(t\right)-\mu_{v}^{\vartheta }I_{v0}\left(t\right)\right], \end{array}\right.\\ \left\{\begin{array}{c} L\left[S_{h12}\left(t\right)\right]=\frac{1}{s^{\vartheta }}L\left[\mu_{h}^{\vartheta }N_{h}-\frac{b^{\vartheta }\beta_{h1}}{N_{h}}D_{1}\left(t\right)-p^{\vartheta }S_{h11}\left(t\right)-\mu_{h}^{\vartheta }S_{h11}\left(t\right)\right],\\ L\left[S_{h22}\left(t\right)\right]=\frac{1}{s^{\vartheta }}L\left[\nu^{\vartheta }R_{h1}\left(t\right)-\frac{b^{\vartheta }\beta_{h2}}{N_{h}}E_{1}\left(t\right)-\mu_{h}^{\vartheta }S_{h21}\left(t\right)\right],\\ L\left[E_{h2}\left(t\right)\right]=\frac{1}{s^{\vartheta }}L\left[\frac{b^{\vartheta }\beta_{h1}}{N_{h}}D_{1}\left(t\right)+\frac{b^{\vartheta }\beta_{h2}}{N_{h}}E_{1}\left(t\right)-\left(\mu_{h}^{\vartheta }+\rho_{h}^{\vartheta }\right)E_{h1}\left(t\right)\right],\\ L\left[I_{h2}\left(t\right)\right]=\frac{1}{s^{\vartheta }}L\left[\left(1-\psi \right)\rho_{h}^{\vartheta }E_{h1}\left(t\right)-\left(\gamma^{\vartheta }+\mu_{h}^{\vartheta }+\tau^{\vartheta }\right)I_{h1}\left(t\right)\right],\\ L\left[I_{hA2}\left(t\right)\right]=\frac{1}{s^{\vartheta }}L\left[\psi \rho_{h}^{\vartheta }E_{h1}\left(t\right)-\left(\gamma^{\vartheta }+\mu_{h}^{\vartheta }\right)I_{hA1}\left(t\right)\right],\\ L\left[R_{h2}\left(t\right)\right]=\frac{1}{s^{\vartheta }}L\left[p^{\vartheta }S_{h11}\left(t\right)+\tau^{\vartheta }I_{h1}\left(t\right)+\gamma^{\vartheta }\left(I_{h1}\left(t\right)+I_{hA1}\left(t\right)\right)-\left(\nu^{\vartheta }+\mu_{h}^{\vartheta }\right)R_{h1}\left(t\right)\right],\\ L\left[S_{v2}\left(t\right)\right]=\frac{1}{s^{\vartheta }}L\left[\mu_{v}^{\vartheta }N_{v}-\frac{b^{\vartheta }\beta_{v}}{N_{h}}F_{1}\left(t\right)-\mu_{v}^{\vartheta }S_{v1}\left(t\right)\right],\\ L\left[E_{v2}\left(t\right)\right]=\frac{1}{s^{\vartheta }}L\left[\frac{b^{\vartheta }\beta_{v}}{N_{h}}F_{1}\left(t\right)-\left(\mu_{v}^{\vartheta }+\rho_{v}^{\vartheta }\right)E_{v1}\left(t\right)\right],\\ L\left[I_{v2}\left(t\right)\right]=\frac{1}{s^{\vartheta }}L\left[\rho_{v}^{\vartheta }E_{v1}\left(t\right)-\mu_{v}^{\vartheta }I_{v1}\left(t\right)\right]. \end{array}\right. \end{array}$$

Furthermore, we attain

(48) $$\begin{array}{c} \left\{\begin{array}{c} L\left[S_{h1\left(j+1\right)}\left(t\right)\right]=\frac{1}{s^{\vartheta }}L\left[\mu_{h}^{\vartheta }N_{h}-\frac{b^{\vartheta }\beta_{h1}}{N_{h}}D_{j}\left(t\right)-p^{\vartheta }S_{h1j}\left(t\right)-\mu_{h}^{\vartheta }S_{h1j}\left(t\right)\right],\\ L\left[S_{h2\left(j+1\right)}\left(t\right)\right]=\frac{1}{s^{\vartheta }}L\left[\nu^{\vartheta }R_{hj}\left(t\right)-\frac{b^{\vartheta }\beta_{h2}}{N_{h}}E_{j}\left(t\right)-\mu_{h}^{\vartheta }S_{h2j}\left(t\right)\right],\\ L\left[E_{h\left(j+1\right)}\left(t\right)\right]=\frac{1}{s^{\vartheta }}L\left[\frac{\beta_{h1}b^{\vartheta }}{N_{h}}D_{j}\left(t\right)+\frac{\beta_{h2}b^{\vartheta }}{N_{h}}E_{j}\left(t\right)-\left(\mu_{h}^{\vartheta }+\rho_{h}^{\vartheta }\right)E_{hj}\left(t\right)\right],\\ L\left[I_{h\left(j+1\right)}\left(t\right)\right]=\frac{1}{s^{\vartheta }}L\left[\left(1-\psi \right)\rho_{h}^{\vartheta }E_{hj}\left(t\right)-\left(\gamma^{\vartheta }+\tau^{\vartheta }+\mu_{h}^{\vartheta }\right)I_{hj}\left(t\right)\right],\\ L\left[I_{hA\left(j+1\right)}\left(t\right)\right]=\frac{1}{s^{\vartheta }}L\left[\psi \rho_{h}^{\vartheta }E_{hj}\left(t\right)-\left(\gamma^{\vartheta }+\mu_{h}^{\vartheta }\right)I_{hAj}\left(t\right)\right],\\ L\left[R_{h\left(j+1\right)}\left(t\right)\right]=\frac{1}{s^{\vartheta }}L\left[p^{\vartheta }S_{h1j}\left(t\right)+\tau^{\vartheta }I_{hj}\left(t\right)+\gamma^{\vartheta }\left(I_{hj}\left(t\right)+I_{hAj}\left(t\right)\right)-\left(\mu_{h}^{\vartheta }+\nu^{\vartheta }\right)R_{hj}\left(t\right)\right],\\ L\left[S_{v\left(j+1\right)}\left(t\right)\right]=\frac{1}{s^{\vartheta }}L\left[\mu_{v}^{\vartheta }N_{v}-\frac{\beta_{v}b^{\vartheta }}{N_{h}}F_{j}\left(t\right)-\mu_{v}^{\vartheta }S_{vj}\left(t\right)\right],\\ L\left[E_{v\left(j+1\right)}\left(t\right)\right]=\frac{1}{s^{\vartheta }}L\left[\frac{b^{\vartheta }\beta_{v}}{N_{h}}F_{j}\left(t\right)-\left(\mu_{v}^{\vartheta }+\rho_{v}^{\vartheta }\right)E_{vj}\left(t\right)\right],\\ L\left[I_{v\left(j+1\right)}\left(t\right)\right]=\frac{1}{s^{\vartheta }}L\left[\rho_{v}^{\vartheta }E_{vj}\left(t\right)-\mu_{v}^{\vartheta }I_{vj}\left(t\right)\right]. \end{array}\right. \end{array}$$

Initial conditions are stated as

(49) $$\begin{array}{c} \left\{\begin{array}{c} S_{h10}\left(t\right)=S_{h10}S_{h20}\left(t\right)=S_{h20},\\ E_{h0}\left(t\right)=E_{h0}I_{h0}\left(t\right)=I_{h0},\\ I_{hA0}\left(t\right)=I_{hA0}R_{h0}\left(t\right)=R_{h0},\\ S_{v0}\left(t\right)=S_{v0}E_{v0}\left(t\right)=E_{v0},\\ I_{v0}\left(t\right)=I_{v0}. \end{array}\right. \end{array}$$

To further simplify it, we proceed as follows:

(50) $$\begin{array}{c} \left\{\begin{array}{c} S_{h11}\left(t\right)=L^{-1}\left[\frac{1}{s^{\vartheta }}L\left[\mu_{h}^{\vartheta }N_{h}-\frac{b^{\vartheta }\beta_{h1}}{N_{h}}D_{0}\left(t\right)-p^{\vartheta }S_{h10}\left(t\right)-\mu_{h}^{\vartheta }S_{h10}\left(t\right)\right]\right],\\ S_{h21}\left(t\right)=L^{-1}\left[\frac{1}{s^{\vartheta }}L\left[\nu^{\vartheta }R_{h0}\left(t\right)-\frac{b^{\vartheta }\beta_{h2}}{N_{h}}E_{0}\left(t\right)-\mu_{h}^{\vartheta }S_{h20}\left(t\right)\right]\right],\\ E_{h1}\left(t\right)=L^{-1}\left[\frac{1}{s^{\vartheta }}L\left[\frac{b^{\vartheta }\beta_{h1}}{N_{h}}A_{0}\left(t\right)+\frac{b^{\vartheta }\beta_{h2}}{N_{h}}E_{0}\left(t\right)-\left(\rho_{h}^{\vartheta }+\mu_{h}^{\vartheta }\right)E_{h0}\left(t\right)\right]\right],\\ I_{h1}\left(t\right)=L^{-1}\left[\frac{1}{s^{\vartheta }}L\left[\left(1-\psi \right)\rho_{h}^{\vartheta }E_{h0}\left(t\right)-\left(\gamma^{\vartheta }+\mu_{h}^{\vartheta }+\tau^{\vartheta }\right)I_{h0}\left(t\right)\right]\right],\\ I_{hA1}\left(t\right)=L^{-1}\left[\frac{1}{s^{\vartheta }}L\left[\psi \rho_{h}^{\vartheta }E_{h0}\left(t\right)-\left(\gamma^{\vartheta }+\mu_{h}^{\vartheta }\right)I_{hA0}\left(t\right)\right]\right],\\ R_{h1}\left(t\right)=L^{-1}\left[\frac{1}{s^{\vartheta }}L\left[p^{\vartheta }S_{h10}\left(t\right)+\tau^{\vartheta }I_{h0}\left(t\right)+\gamma^{\vartheta }\left(I_{h0}\left(t\right)+I_{hA0}\left(t\right)\right)-\left(\mu_{h}^{\vartheta }+\nu^{\vartheta }\right)R_{h0}\left(t\right)\right]\right],\\ S_{v1}\left(t\right)=L^{-1}\left[\frac{1}{s^{\vartheta }}L\left[\mu_{v}^{\vartheta }N_{v}-\frac{b^{\vartheta }\beta_{v}}{N_{h}}F_{0}\left(t\right)-\mu_{v}^{\vartheta }S_{v0}\left(t\right)\right]\right],\\ E_{v1}\left(t\right)=L^{-1}\left[\frac{1}{s^{\vartheta }}L\left[\frac{b^{\vartheta }\beta_{v}}{N_{h}}F_{0}\left(t\right)-\left(\mu_{v}^{\vartheta }+\rho_{v}^{\vartheta }\right)E_{v0}\left(t\right)\right]\right],\\ I_{v1}\left(t\right)=L^{-1}\left[\frac{1}{s^{\vartheta }}L\left[\rho_{v}^{\vartheta }E_{v0}\left(t\right)-\mu_{v}^{\vartheta }I_{v0}\left(t\right)\right]\right], \end{array}\right.\\ \left\{\begin{array}{c} S_{h12}\left(t\right)=L^{-1}\left[\frac{1}{s^{\vartheta }}L\left[\mu_{h}^{\vartheta }N_{h}-\frac{b^{\vartheta }\beta_{h1}}{N_{h}}D_{1}\left(t\right)-p^{\vartheta }S_{h11}\left(t\right)-\mu_{h}^{\vartheta }S_{h11}\left(t\right)\right]\right],\\ S_{h22}\left(t\right)=L^{-1}\left[\frac{1}{s^{\vartheta }}L\left[\nu^{\vartheta }R_{h1}\left(t\right)-\frac{b^{\vartheta }\beta_{h2}}{N_{h}}E_{1}\left(t\right)-\mu_{h}^{\vartheta }S_{h21}\left(t\right)\right]\right],\\ E_{h2}\left(t\right)=L^{-1}\left[\frac{1}{s^{\vartheta }}L\left[\frac{b^{\vartheta }\beta_{h1}}{N_{h}}D_{1}\left(t\right)+\frac{b^{\vartheta }\beta_{h2}}{N_{h}}E_{1}\left(t\right)-\left(\rho_{h}^{\vartheta }+\mu_{h}^{\vartheta }\right)E_{h1}\left(t\right)\right]\right],\\ I_{h2}\left(t\right)=L^{-1}\left[\frac{1}{s^{\vartheta }}L\left[\rho_{h}^{\vartheta }\left(1-\psi \right)E_{h1}\left(t\right)-\left(\gamma^{\vartheta }+\mu_{h}^{\vartheta }+\tau^{\vartheta }\right)I_{h1}\left(t\right)\right]\right],\\ I_{hA2}\left(t\right)=L^{-1}\left[\frac{1}{s^{\vartheta }}L\left[\rho_{h}^{\vartheta }\psi E_{h1}\left(t\right)-\left(\gamma^{\vartheta }+\mu_{h}^{\vartheta }\right)I_{hA1}\left(t\right)\right]\right],\\ R_{h2}\left(t\right)=L^{-1}\left[\frac{1}{s^{\vartheta }}L\left[p^{\vartheta }S_{h11}\left(t\right)+\tau^{\vartheta }I_{h1}\left(t\right)+\gamma^{\vartheta }\left(I_{h1}\left(t\right)+I_{hA1}\left(t\right)\right)-\left(\mu_{h}^{\vartheta }+\nu^{\vartheta }\right)R_{h1}\left(t\right)\right]\right],\\ S_{v2}\left(t\right)=L^{-1}\left[\frac{1}{s^{\vartheta }}L\left[\mu_{v}^{\vartheta }N_{v}-\frac{b^{\vartheta }\beta_{v}}{N_{h}}F_{1}\left(t\right)-\mu_{v}^{\vartheta }S_{v1}\left(t\right)\right]\right],\\ E_{v2}\left(t\right)=L^{-1}\left[\frac{1}{s^{\vartheta }}L\left[\frac{b^{\vartheta }\beta_{v}}{N_{h}}F_{1}\left(t\right)-\left(\mu_{v}^{\vartheta }+\rho_{v}^{\vartheta }\right)E_{v1}\left(t\right)\right]\right],\\ I_{v2}\left(t\right)=L^{-1}\left[\frac{1}{s^{\vartheta }}L\left[\rho_{v}^{\vartheta }E_{v1}\left(t\right)-\mu_{v}^{\vartheta }I_{v1}\left(t\right)\right]\right]. \end{array}\right. \end{array}$$

Furthermore, we get that

(51) $$\begin{array}{c} \left\{\begin{array}{c} S_{h1\left(j+1\right)}\left(t\right)=L^{-1}\left[\frac{1}{s^{\vartheta }}L\left[\mu_{h}^{\vartheta }N_{h}-\frac{b^{\vartheta }\beta_{h1}}{N_{h}}D_{j}\left(t\right)-p^{\vartheta }S_{h1j}\left(t\right)-\mu_{h}^{\vartheta }S_{h1j}\left(t\right)\right]\right],\\ S_{h2\left(j+1\right)}\left(t\right)=L^{-1}\left[\frac{1}{s^{\vartheta }}L\left[\nu^{\vartheta }R_{hj}\left(t\right)-\frac{b^{\vartheta }\beta_{h2}}{N_{h}}E_{j}\left(t\right)-\mu_{h}^{\vartheta }S_{h2j}\left(t\right)\right]\right],\\ E_{h\left(j+1\right)}\left(t\right)=L^{-1}\left[\frac{1}{s^{\vartheta }}L\left[\frac{\beta_{h1}b^{\vartheta }}{N_{h}}A_{j}\left(t\right)+\frac{b^{\vartheta }\beta_{h2}}{N_{h}}B_{j}\left(t\right)-\left(\rho_{h}^{\vartheta }+\mu_{h}^{\vartheta }\right)E_{hj}\left(t\right)\right]\right],\\ I_{h\left(j+1\right)}\left(t\right)=L^{-1}\left[\frac{1}{s^{\vartheta }}L\left[\left(1-\psi \right)\rho_{h}^{\vartheta }E_{hj}\left(t\right)-\left(\gamma^{\vartheta }+\mu_{h}^{\vartheta }+\tau^{\vartheta }\right)I_{hj}\left(t\right)\right]\right],\\ I_{hA\left(j+1\right)}\left(t\right)=L^{-1}\left[\frac{1}{s^{\vartheta }}L\left[\psi \rho_{h}^{\vartheta }E_{hj}\left(t\right)-\left(\gamma^{\vartheta }+\mu_{h}^{\vartheta }\right)I_{hAj}\left(t\right)\right]\right],\\ R_{h\left(j+1\right)}\left(t\right)=L^{-1}\left[\frac{1}{s^{\vartheta }}L\left[p^{\vartheta }S_{h1j}\left(t\right)+\tau^{\vartheta }I_{hj}\left(t\right)+\gamma^{\vartheta }\left(I_{hj}\left(t\right)+I_{hAj}\left(t\right)\right)-\left(\mu_{h}^{\vartheta }+\nu^{\vartheta }\right)R_{hj}\left(t\right)\right]\right],\\ S_{v\left(j+1\right)}\left(t\right)=L^{-1}\left[\frac{1}{s^{\vartheta }}L\left[\mu_{v}^{\vartheta }N_{v}-\frac{b^{\vartheta }\beta_{v}}{N_{h}}F_{j}\left(t\right)-\mu_{v}^{\vartheta }S_{vj}\left(t\right)\right]\right],\\ E_{v\left(j+1\right)}\left(t\right)=L^{-1}\left[\frac{1}{s^{\vartheta }}L\left[\frac{b^{\vartheta }\beta_{v}}{N_{h}}F_{j}\left(t\right)-\left(\mu_{v}^{\vartheta }+\rho_{v}^{\vartheta }\right)E_{vj}\left(t\right)\right]\right],\\ I_{v\left(j+1\right)}\left(t\right)=L^{-1}\left[\frac{1}{s^{\vartheta }}L\left[\rho_{v}^{\vartheta }E_{vj}\left(t\right)-\mu_{v}^{\vartheta }I_{vj}\left(t\right)\right]\right]. \end{array}\right. \end{array}$$

Therefore, we have the following answer in series form:

(52) $$\begin{array}{c} \left\{\begin{array}{c} S_{v}\left(t\right)=S_{v0}\left(t\right)+S_{v1}\left(t\right)+S_{v2}\left(t\right)+S_{v3}\left(t\right)+\cdots ,\\ E_{v}\left(t\right)=E_{v0}\left(t\right)+E_{v1}\left(t\right)+E_{v2}\left(t\right)+E_{v3}\left(t\right)+\cdots ,\\ I_{v}\left(t\right)=I_{v0}\left(t\right)+I_{v1}\left(t\right)+I_{v2}\left(t\right)+I_{v3}\left(t\right)+\cdots ,\\ S_{h1}\left(t\right)=S_{h10}\left(t\right)+S_{h11}\left(t\right)+S_{h12}\left(t\right)+S_{h13}\left(t\right)+\cdots ,\\ S_{h2}\left(t\right)=S_{h20}\left(t\right)+S_{h21}\left(t\right)+S_{h22}\left(t\right)+S_{h23}\left(t\right)+\cdots ,\\ E_{h}\left(t\right)E_{h0}\left(t\right)+E_{h1}\left(t\right)+E_{h2}\left(t\right)+E_{h3}\left(t\right)+\cdots ,\\ I_{h}\left(t\right)=I_{h0}\left(t\right)+I_{h1}\left(t\right)+I_{h2}\left(t\right)+I_{h3}\left(t\right)+\cdots ,\\ I_{hA}\left(t\right)=I_{hA0}\left(t\right)+I_{hA1}\left(t\right)+I_{hA2}\left(t\right)+I_{hA3}\left(t\right)+\cdots ,\\ R_{h}\left(t\right)R_{h0}\left(t\right)+R_{h1}\left(t\right)+R_{h2}\left(t\right)+R_{h3}\left(t\right)+\cdots . \end{array}\right. \end{array}$$

The upper mentioned numerical technique is utilized to investigate the dynamics (8) of dengue infection. For numerical reasons, the parameter values in Table 1 are utilized. Here, we will perform distinct numerical scenario to illustrate the impact of input factors on the system of dengue. As a result of our findings, we will recommend effective control strategies that will minimize the frequency of dengue fever in population. Using simulations, we showed the time series of infected, exposed, and asymptotic carriers in the host population, while we emphasized the time series of exposed and diseased people in the vector population.

The article "Qualitative Analysis of the Transmission Dynamics of Dengue with the Effect of Memory, Reinfection, and Vaccination" was published in 2022. Journal: Comput Math Methods Med.

The influence of vaccination on dengue transmission patterns has been depicted in the first simulation shown in Figure 1. The human and mosquito time series are indicated with varied vaccination *p* values. It has been discovered that vaccination can reduce the degree of infection; hence, it is advised that vaccine efficacy be improved in order to eliminate dengue infection. In Figure 2, we highlighted the influence of treatment *τ* on the system of dengue in the second simulation. We proposed that therapy can be utilized as a control parameter to minimize infection levels in society. The role of mosquito bite rate is depicted in Figure 3 which illustrated that the biting rate is vital and can transmit the illness; therefore, controlling this aspect is crucial to avoid infection transmission.

The effect of the asymptotic carrier on the system is seen in the fourth scenario in Figure 4. It was demonstrated that this input component is crucial and can be a source of infection in dengue-endemic locations. In Figure 5, the role of the losing rate of immunity *ν* has been visualised. This parameter is equally harmful, as shown by the results, and can enable dengue process more complicated. In Figure 6, we graphically represented the influence of memory on the time series of dengue infection. The plot of the infected individuals was illustrated with various values of memory *ϑ*. This parameter seems to be effective and recommended to the policymakers for better control of the infection.

Memory plays a crucial part in vector-borne disease transmission dynamics because vector-borne sickness has knowledge of previous stages and an associative learning experience [15, 16]. In dengue transmission, mosquitoes use their prior experience about the human's location, blood selection, colour, and the smell of humans sweat to reduce the contact rate between vector and hosts. Fractional-order models give information about the past and present states of biological systems for the future. Moreover, fractional-order models possess hereditary properties and represent the nonlocal behavior of biological systems. Therefore, the results of fractional models are more accurate than that of integer models, and the index of memory may be utilized as a control measure. Fractional-order systems may readily reflect these kinds of phenomena in mathematical models of infectious diseases. As a result, it is crucial to consider memory's role in the spread of dengue disease. We primarily focused on such elements in our study to demonstrate their influence on infection dynamics. Our findings showed that the memory index can limit infection levels, which is something policymakers should consider. We proved that vaccination and diagnosis can help to stabilize dengue fever and the index of memory may be utilized as a control measure.

The article "Qualitative Analysis of the Transmission Dynamics of Dengue with the Effect of Memory, Reinfection, and Vaccination" was published in 2022. Journal: Comput Math Methods Med.

## 7. Conclusion

Dengue fever is a life-threatening and severe sickness that affects people all over the globe. Introducing effective techniques for the management of this viral infection is now a problem for policymakers, scientists, and public health professionals. Through a fractional framework, we developed a new for dengue fever that includes asymptotic carriers, immunisation, reinfection, and therapy. With the use of the fixed-point theorem, the existence and uniqueness of the solution of the hypothesized system are explored in the context of Banach's and Schaefer's. We created the necessary parameters for the Ulam-Hyers stability in our dengue system. The effect of various variables on the dynamics of dengue is evaluated using the LADM approach to describe the effect of various input factors on the time series of dengue. We found that biting rates, asymptomatic carriers, and immunity loss rates are significant characteristics that make control more challenging, but dengue infection can be eliminated by vaccine, memory index, and therapy. We demonstrated the impact of memory on the time series of dengue and proposed that it may be employed as a control parameter for infection management. We shall demonstrate the influence of incubation and maturation delay on dengue transmission in future studies.

## Figures and Tables

**Figure 1:** Graphical view analysis of system (8) with distinct values of *p*, i.e., *p* = 0.535, 0.435, 0.335, and 0.235, for dengue dynamics.

**Figure 2:** Graphical view analysis of system (8) distinct values of *τ*, i.e., *τ* = 0.040, 0.035, 0.30, and 0.025, for dengue dynamics.

**Figure 3:** Plotting the time series of the system (8) with distinct values of *b*, i.e., *b* = 0.55, 0.50, 0.45, and 0.40, for dengue dynamics.

**Figure 4:** Representation of the system (8) with distinct values of the input factor *ψ*, i.e., *ψ* = 0.7, 0.6, 0.5, and 0.4, for dengue fever.

**Figure 5:** Plotting the time series of the system (8) with distinct values of *ν*, i.e., *ν* = 0.005, 0.010, 0.015, and 0.020, for dengue fever.

**Figure 6:** Plotting of the system (8) with distinct values of memory, i.e., *ϑ* = 1.0, 0.9, 0.8, and 0.7, for dengue fever.

**Table 1:** In numerical analysis, the values of input parameters with descriptions are used.

Input factors	Interpretations	Values	Reference
*μ*_*h*_	Natural fatality and birth frequency of humans	0.000046 and 0.004500	[31]
*β*_*v*_	Transmission probability from hosts to vectors	0.75	[11]
*τ*	Treatment rate of humans	0.5	Supposed
*ν*	The rate at which humans loss immunity	0.05	Supposed
*b*	Vectors biting frequency	0.5	[11]
*ψ*	Asymptomatic fraction of infected individuals	0.6	Supposed
*β*_*h*1_	The rate at which mosquitoes are transferred to *S*_*h*1_	0.75	[11]
*β*_*h*2_	The rate at which mosquitoes are transferred to *S*_*h*2_	0.375	Supposed
*p*	Fraction of susceptible *S*_*h*1_ that is vaccinated	0.3	Supposed
*γ*	Recovery rate of host	0.3288330	[31]
*μ*_*v*_	Natural fatality and birth frequency of mosquitoes	0.032300 and 0.029410	[31]
*ϑ*	Fractional order	0.6	Assume

The article "Qualitative Analysis of the Transmission Dynamics of Dengue with the Effect of Memory, Reinfection, and Vaccination" was published in 2022. Journal: Comput Math Methods Med.

## Data Availability

The data that support the findings of this study are available from the corresponding author upon reasonable request.
